The article "Development and Validation of Diagnostic Models for Hand-Foot-and-Mouth Disease in Children" was retracted in 2023. Reasons: unreliable results or conclusions; concerns about the data; concerns about the peer review; concerns about the citations.

# Development and Validation of Diagnostic Models for Hand-Foot-and-Mouth Disease in Children

**DOI:** 10.1155/2021/1923636

**Published:** 2021-08-30

**Authors:** Feng Zhuo, Mengjie Yu, Qiang Chen, Nuoya Li, Li Luo, Meiying Hu, Qi Dong, Liang Hong, Shouhua Zhang, Qiang Tao

**Affiliations:** ^1^Pediatric Cardiology Center, Jiangxi Provincial Children's Hospital, Nanchang, Jiangxi 330006, China; ^2^Key Laboratory of Drug Metabolism and Pharmacokinetics, China Pharmaceutical University, Nanjing, 210009 Jiangsu, China; ^3^Department of Respiratory, Jiangxi Provincial Children's Hospital, Nanchang, Jiangxi 330006, China; ^4^Department of General Surgery, Jiangxi Provincial Children's Hospital, Nanchang, Jiangxi 330006, China; ^5^Department of General Surgery, The Affiliated Children's Hospital of Nanchang University, Nanchang, Jiangxi 330006, China

## Abstract

**Objective:**

To find risk markers and develop new clinical predictive models for the differential diagnosis of hand-foot-and-mouth disease (HFMD) with varying degrees of disease.

**Methods:**

19766 children with HFMD and 64 clinical indexes were included in this study. The patients included in this study were divided into the mild patients' group (mild) with 12292 cases, severe patients' group (severe) with 6508 cases, and severe patients with respiratory failure group (severe-RF) with 966 cases. Single-factor analysis was carried out on 64 indexes collected from patients when they were admitted to the hospital, and the indexes with statistical differences were selected as the prediction factors. Binary multivariate logistic regression analysis was used to construct the prediction models and calculate the adjusted odds ratio (OR).

**Results:**

SP, DP, NEUT#, NEUT%, RDW-SD, RDW-CV, GGT, CK/CK-MB, and Glu were risk markers in mild/severe, mild/severe-RF, and severe/severe-RF. Glu was a diagnostic marker for mild/severe-RF (AUROC = 0.80, 95% CI: 0.78-0.82); the predictive model constructed by temperature, SP, MOMO%, EO%, RDW-SD, GLB, CRP, Glu, BUN, and Cl could be used for the differential diagnosis of mild/severe (AUROC > 0.84); the predictive model constructed by SP, age, NEUT#, PCT, TBIL, GGT, Mb, *β*2MG, Glu, and Ca could be used for the differential diagnosis of severe/severe-RF (AUROC > 0.76).

**Conclusion:**

By analyzing clinical indicators, we have found the risk markers of HFMD and established suitable predictive models.

## 1. Introduction

Hand-foot-and-mouth disease (HFMD) is a common viral illness mainly caused by enterovirus 71 (EV71) and coxsackie A16 (CA16), which mainly affects children under 5 years of age [1, 2]. Most patients with HFMD have mild symptoms and can be cured in 7-10 days. However, a small number of patients will get worse and may have serious complications, such as nervous system damage and cardiopulmonary failure, which will lead to death [3, 4]. Early detection of severe HFMD with the worsening condition and timely appropriate treatment and nursing can significantly improve the treatment and prognosis of the children [5, 6]. Therefore, it is particularly important to develop a clinical decision-making tool to predict and early identify HFMD patients with different degrees of disease to provide effective interventions.

The article "Development and Validation of Diagnostic Models for Hand-Foot-and-Mouth Disease in Children" was retracted in 2023. Reasons: unreliable results or conclusions; concerns about the data; concerns about the peer review; concerns about the citations.

Although many previous studies have focused on investigating the risk markers and exploring prediction models of HFMD [7–10], there are still few studies to find the risk factors of HFMD patients and establish a prediction model by using only various laboratory test indicators. In this study, retrospective case-control analysis was used to explore the risk factors of early recognition of progression from mild to severe and from common severe to severe-RF by analyzing various types of blood test indicators of HFMD patients with different degrees of illness; to establish a suitable risk prediction model to objectively, systematically, and quantitatively evaluate the patient's condition; to explore the possibility of early progression of HFMD to severe and common severe to severe-RF; and to take early intervention measures, guide clinical treatment, and reduce the mortality of patients.

## 2. Methods

### 2.1. Participating Cohorts

From April 2009 to January 2020, patients with HFMD admitted to Jiangxi Children's Hospital were selected as the study objects, and the definition diagnosis of HFMD was based on the guidelines for the diagnosis and treatment of hand-foot-and-mouth disease (http://www.nhc.gov.cn/wjw/gfxwj/201304/4a5c8d7485c64d189afd5392a390bd84.shtml/; http://www.nhc.gov.cn/yzygj/wslgf/201306/6d935c0f43cd4a1fb46f8f71acf8e245.shtml/; http://www.nhc.gov.cn/yzygj/s3594q/201805/5db274d8697a41ea84e88eedd8bf8f63.shtml/). Inclusion criteria were positive enterovirus-specific nucleic acid test (CV-A16, EV-A71, etc.) or isolated enterovirus and identified as CV-A16, EV-A71, or other enterovirus causing HFMD. We also excluded several children with erupting diseases (e.g., papular urticaria, sandskin rash, chickenpox, atypical measles, infantile rash, shingles, rubella, and bullous rash caused by CV-A16 or EV-A71). The data used in this study were all detected at the first visit of patients. This retrospective study was approved by the ethics committee of Jiangxi Provincial Children's Hospital.

### 2.2. Outcomes

The categories of diagnosis results are mild, severe, and severe-RF, which mainly refer to the guidelines for the diagnosis and treatment of hand-foot-and-mouth disease. The main symptoms of mild patients are fever and rash of hands, feet, mouth, buttocks, and other parts, which can be accompanied by cough, runny nose, anorexia, and other symptoms. Some cases only present as rash or herpetic pharyngitis, and some cases may be without rash. Typical rashes are maculopapules, papules, and herpes. There is inflammatory redness around the rash, less fluidity in herpes, no pain, no itching, no scabs, and no scars when the rash recovers. Atypical rashes are usually small, thick, hard, and few, sometimes with ecchymosis. Some types of enteroviruses, such as CV-A6 and CV-A10, cause severe skin lesions, and the rash may present as bulla-like changes with pain and itching, not limited to the hands, feet, and mouth.

The article "Development and Validation of Diagnostic Models for Hand-Foot-and-Mouth Disease in Children" was retracted in 2023. Reasons: unreliable results or conclusions; concerns about the data; concerns about the peer review; concerns about the citations.

The main manifestations of severe patients are central nervous system damage, which usually occurs within 1-5 days of the course of the disease. The manifestations are mental illness, drowsiness, weakness of sucking, easily frightened, headache, vomiting, fidgety, limb shaking, myasthenia, neck rigidity, etc. Patients with severe respiratory failure were mainly characterized by increased heart rate and respiration, cold sweat, cold extremities, flowy skin, elevated blood pressure or tachycardia (bradycardia in some children), tachycardia, cyanosis of the mouth, coughing pink foaming sputum or bloody fluid, decreased blood pressure, or shock. All data were collected independently of the evaluation of the study results.

### 2.3. Variables and Statistical Analysis

Gender, age, clinical blood test indicators, and other information collected at the first visit of HFMD patients were taken as potential predictive variables, and cases with blood test indicators missing more than 30% and variables with data missing more than 10% were eliminated. The processing method of missing values in the data was as follows: mode was used for interpolation of classified variables and mean was used for interpolation of continuous variables. For variables that do not conform to the normal distribution, the Mann–Whitney *U* test was used, and for variables that conform to the normal distribution, the independent-sample *t*-test was used. A *P* value < 0.05 was regarded as being statistically significant for all of the analyses. The adjusted odds ratio (OR) of each variable was obtained by logistic regression analysis. To estimate the ability to discriminate between patients with different diagnoses, we used the receiver operating characteristic (ROC) curve analysis for pairs of patients [11]. All analyses were performed using R software (version 4.0) and SPSS 26.0 (SPSS Inc., Chicago, IL, US).

The article "Development and Validation of Diagnostic Models for Hand-Foot-and-Mouth Disease in Children" was retracted in 2023. Reasons: unreliable results or conclusions; concerns about the data; concerns about the peer review; concerns about the citations.

## 3. Results

### 3.1. Study Population

Generally, 19766 children with HFMD met the inclusion criteria of this study, and 3091 children were excluded. The patients included in this study were divided into the mild patients' group (mild) with 12292 cases, severe patients' group (severe) with 6508 cases, and severe patients with respiratory failure group (severe-RF) with 966 cases. 64 predictive variables met the requirements and 24 variables were excluded. Some basic information and information on variables of subjects in each group are shown in Table 1.

### 3.2. Screening and Analysis of Difference Indexes

Through the statistical analysis of all the indicators included in the study, we found that 52, 44, and 51 indicators showed statistical differences between mild/severe, severe/severe-RF, and mild/severe-RF, respectively, and 30 indicators showed significant differences among the three groups (Table 2). With the aggravation of patients' condition, 23 indicators showed a significant trend of change (Table 2). The contents of 10 indicators including SP, DP, NEUT#, NEUT%, RDW-SD, RDW-CV, GGT, LDH, CK/CK-MB, and Glu showed an increasing trend in the blood of mild, severe, and severe-RF patients, while those of 13 indicators presented a decreasing trend, including LYMPH%, MONO%, EO#, EO%, BASO%, MCHC, ALB, ALB/GLB, *β*2MG, CRP, K, Na, and Cl.

### 3.3. Analysis of Risk Factors

Calculating the adjusted OR values between the mild/severe, mild/severe-RF, and severe/severe-RF groups, we found that a total of 19 indicators may be risk factors of mild development to severe (adjusted OR > 1.0), where temperature (adjusted OR = 2.76, 95% CI: 2.66-2.86) and Glu (adjusted OR = 1.60, 95% CI: 1.55-1.64) performed better (Figure 1(a)). A total of 17 indicators may be risk factors of mild development to severe-RF (adjusted OR > 1.0), among which temperature (adjusted OR = 2.67, 95% CI: 2.48-2.88) and Glu (adjusted OR = 1.75, 95% CI: 1.67-1.83) performed better (Figure 1(b)). A total of 13 indicators may be risk factors of severe development to severe-RF (adjusted OR > 1.0), of which Glu (adjusted OR = 1.22, 95% CI: 1.17-1.27) performed best (Figure 1(c)). We further analyzed and found that 9 indicators of SP, DP, NEUT#, NEUT%, RDW-SD, RDW-CV, GGT, CK/CK-MB, and Glu can be used as risk factors in mild/severe, mild/severe-RF, and severe/severe-RF. And with the aggravation of HFMD patients, the levels of these 9 indicators in the blood of mild, severe, and severe-RF patients all showed a significant increasing trend (Figure 2). Therefore, we speculate that these 9 indicators might be risk factors for HFMD and played an important role in suggesting the aggravation of patients' condition.

The article "Development and Validation of Diagnostic Models for Hand-Foot-and-Mouth Disease in Children" was retracted in 2023. Reasons: unreliable results or conclusions; concerns about the data; concerns about the peer review; concerns about the citations.

### 3.4. ROC Analysis of Difference Indexes

ROC curve analysis was used to investigate the diagnostic performance of each difference indicator. The top 10 indicators with good performance among each group are shown in Table 3. The results show that Glu (AUROC = 0.80, 95% CI: 0.78-0.82) can distinguish mild from severe-RF well. However, in mild/severe and severe/severe-RF, the single index does not differentiate well (AUROC < 0.75).

### 3.5. Development and Validation of Prediction Models

To improve the diagnostic distinction effect between mild/severe and severe/severe-RF, we further established prediction models. Two-thirds of the participants were randomly assigned to the model development data set, and one-third was kept as the independent validation data set. The variables with significant differences in mild/severe and severe/severe-RF were used as the prediction variables, and binary logistic regression analysis was used to establish the prediction models. The inclusion criterion of model variables was the Akaike Information Criterion (AIC) [12], and stepwise regression was used to fit the best logistic regression model. Because the variables with significant differences between mild/severe and severe/severe-RF were inconsistent, the prediction variables included in the final two models were different.

For the mild and severe groups, 10 indicators of temperature, SP, MOMO%, EO%, RDW-SD, GLB, CRP, Glu, BUN, and Cl were selected in this study to establish a prediction model, and the model equation was *P* = exp(*K*)/(1 + exp(*K*)) and *K* = 0.987 × temperature + 0.026 × SP − 0.073 × MOMO% − 0.291 × EO% + 0.089 × RDW − SD + 0.061 × GLB − 0.020 × CRP + 0.279 × Glu − 0.213 × BUN − 0.096 × Cl − 34.858; *P* > 0.5 was identified as a severe patient. Finally, in the model development data set, the AUROC was 0.845 (95% CI: 0.838-0.852) and the sensitivity and specificity were 72.19% and 81.84%, respectively (Figure 3(a)), and in the validation data set, the AUROC was 0.839 (95% CI: 0.829-0.850) and the sensitivity and specificity were 72.00% and 81.52%, respectively (Figure 3(b)).

For the severe and severe-RF groups, SP, age, NEUT#, PCT, TBIL, GGT, Mb, *β*2MG, Glu, and Ca10 were selected to establish the prediction model, and the model equation was *P* = exp(*K*)/(1 + exp(*K*)), *K* = 0.047 × SP − 0.001 × age + 0.078 × NEUT#+2.621 × PCT − 0.068 × TBIL + 0.013 × GGT + 0.013 × Mb − 0.705 × *β*2MG + 0.154 × Glu − 2.060 × Ca − 1.790; *P* > 0.5 was identified as severe-RF patients. Finally, in the model development data set, the AUROC was 0.766 (95% CI: 0.745-0.786) and the sensitivity and specificity were 59.08% and 80.70%, respectively (Figure 3(c)), and in the validation data set, the AUROC was 0.776 (95% CI: 0.747-0.806) and the sensitivity and specificity were 78.20% and 62.98%, respectively (Figure 3(d)).

The article "Development and Validation of Diagnostic Models for Hand-Foot-and-Mouth Disease in Children" was retracted in 2023. Reasons: unreliable results or conclusions; concerns about the data; concerns about the peer review; concerns about the citations.

## 4. Discussion

Severe HFMD patients have an acute onset and serious condition, often accompanied by serious complications (such as nervous system damage and cardiopulmonary failure), which will lead to death [3, 4]. Therefore, it is of great significance to find appropriate risk factors for early intervention and treatment of severe HFMD patients.

We analyzed the clinical data of patients with HFMD and found that temperature and Glu performed the best for warning of mild development into severe and severe-RF, and Glu performed the best for warning of severe development and severe-RF. Also, temperature and Glu as risk factors for HFMD have been reported in many pieces of literature [8, 13–15]. In the further analysis of the risk factors between each group, we found that the content of SP, DP, NEUT#, NEUT%, RDW-SD, RDW-CV, GGT, CK/CK-MB, and Glu 9 indicators in mild, severe, and severe-RF patients all showed a significant increasing trend and can be used as risk factors in mild/severe, mild/severe-RF, and severe/severe-RF. Peng et al. found that in patients with severe HFMD, hyperglycemia, hypertension, and tachycardia are risk factors for neurogenic pulmonary edema [14]. Fang et al. also found that increased neutrophil count and increased EV71 infection are risk factors for severe HFMD [15]. Therefore, we speculate that these 9 indicators are closely related to the progression of HFMD patients and are potential risk predictors of HFMD. In the follow-up study, we will use these indicators as predictors to build a risk prediction model and subdivide and quantify the risks of each type of HFMD.

Although China has issued diagnosis and treatment guidelines for HFMD, scholars have established various prediction models based on local climate conditions, seasons, and other information [16–18], using the clinical prediction rules (CPRs) [19], machine learning system [20], and other conditions, but no relevant reports have been reported on the diagnosis of mild, severe, and severe-RF by clinical detection. In this study, we found that Glu performs better in the differential diagnosis of mild/severe-RF, and then, we developed and validated clinical prediction models for mild/severe and severe/severe-RF, respectively. The ROC curve showed that the models had good discrimination and accuracy, which could be used to diagnose HFMD patients with different conditions. Compared with the prediction models, CPRs [19], machine learning system [20], and nomogram [7] developed based on information such as climatic conditions and seasons, the indicators used in our model are all derived from patients and are more closely related to HFMD patients. It is more suitable for clinical diagnosis.

The article "Development and Validation of Diagnostic Models for Hand-Foot-and-Mouth Disease in Children" was retracted in 2023. Reasons: unreliable results or conclusions; concerns about the data; concerns about the peer review; concerns about the citations.

During the development of the model, we tried to build a model with the indicators of significant differences between the mild/severe and severe/severe-RF groups as the predictive variables to differentiate and diagnose the mild/severe and severe/severe-RF at the same time, but the discrimination was not good. For example, the temperature has a significant difference in mild/severe, but no difference in severe/severe-RF. However, when developing the prediction model of mild/severe, there is a large difference in the AUROC of whether to include temperature in the model built for prediction variables (included/excluded = 0.845/0.802). Temperature is not included here, and the modeling data is only obtained during model development and no detailed data is provided in this paper. The severity of disease of mild, severe, and severe-RF is different, and the importance of different predictive variables in establishing the prediction model of mild/severe and severe/severe-RF is different. Therefore, we chose different prediction factors for mild/severe and severe/severe-RF to build two different prediction models.

## 5. Strengths and Limitations of This Study

The advantage of our study is that, compared with the existing literature reports, the number of cases included in this study is more (19766 cases), covering mild, severe, and severe-RF patients, and for the first time, blood test indicators are used to establish the prediction model of severe and severe-RF. The limitations of this study, the lack of virus types in the data leading to HFMD, may lead to bias and limit clinical practice. Moreover, this study is a single-center retrospective study conducted in Jiangxi Province, China. We are not sure whether our results can show similar results in other ethnic groups in other regions. Finally, some qualitative indicators (such as lethargy, hyperglycemia, and vomiting) also play a certain role in the diagnosis of HFMD with different conditions, but this study is not included. In the follow-up study, we will investigate whether combining these indicators will optimize our model.

## 6. Conclusion

For the HFMD patients with mild, severe, and severe-RF, we have found appropriate risk factors and developed appropriate predictive models to help clinicians diagnose severe and severe-RF HFMD patients early.

## Figures and Tables

**Figure 1:** Risk factors of mild/severe, mild/severe-RF, and severe/severe-RF.

**Figure 2:** Changes in the content of 9 risk factors.

The article "Development and Validation of Diagnostic Models for Hand-Foot-and-Mouth Disease in Children" was retracted in 2023. Reasons: unreliable results or conclusions; concerns about the data; concerns about the peer review; concerns about the citations.

**Figure 3:** ROC curve of prediction model of mild/severe and severe/severe-RF in development queue and verification queue.

**Table 1:** General characteristics of included populations.

Characteristics	Mild	Severe	Severe-RF
Num	12292	6508	966
Male	8152	4353	673
Age (days)	664.12 ± 4.66	670.56 ± 4.61	643.81 ± 10.99
Weight (kg)	11.34 ± 0.03	11.25 ± 0.03	11.40 ± 0.41
Temperature (°C)	37.41 ± 0.01	38.20 ± 0.01	38.18 ± 0.03
SP (mmHg)	90.91 ± 0.07	94.15 ± 0.12	100.29 ± 0.43
DP (mmHg)	54.01 ± 0.07	57.00 ± 0.11	60.50 ± 0.38
NEUT# (×10^9^/L)	6.67 ± 0.04	7.11 ± 0.05	9.03 ± 0.16
NEUT% (%)	51.33 ± 0.15	57.19 ± 0.20	63.52 ± 0.51
LYMPH# (×10^9^/L)	4.56 ± 0.02	4.09 ± 0.03	4.03 ± 0.10
LYMPH% (%)	38.17 ± 0.14	34.28 ± 0.17	29.36 ± 0.46
MONO# (×10^9^/L)	1.16 ± 0.01	0.94 ± 0.01	0.90 ± 0.02
MONO% (%)	9.26 ± 0.03	7.80 ± 0.05	6.70 ± 0.11
EO# (×10^9^/L)	0.12 ± 0.00	0.06 ± 0.00	0.04 ± 0.00
EO% (%)	1.12 ± 0.01	0.49 ± 0.01	0.29 ± 0.02
BASO# (×10^9^/L)	0.02 ± 0.00	0.02 ± 0.00	0.01 ± 0.00
BASO% (%)	0.15 ± 0.00	0.13 ± 0.00	0.09 ± 0.01
WBC (×10^9^/L)	12.54 ± 0.05	12.22 ± 0.05	14.05 ± 0.20
RBC (×10^12^/L)	4.53 ± 0.00	4.56 ± 0.00	4.56 ± 0.01
HGB (g/L)	116.67 ± 0.09	116.67 ± 0.12	114.82 ± 0.36
MCH (pg)	25.89 ± 0.03	25.86 ± 0.03	25.62 ± 0.07
MCHC (g/L)	327.29 ± 0.27	325.32 ± 0.20	322.61 ± 0.49
RDW-SD (fL)	39.55 ± 0.03	40.34 ± 0.04	41.00 ± 0.11
HCT (%)	35.70 ± 0.03	35.90 ± 0.04	35.64 ± 0.11
MCV (fL)	79.11 ± 0.05	79.60 ± 0.07	79.40 ± 0.19
PLT (×10^9^/L)	300.98 ± 0.86	301.81 ± 1.13	331.52 ± 3.36
P-LCR (%)	27.29 ± 0.07	25.96 ± 0.09	25.87 ± 0.23
MPV (fL)	10.31 ± 0.01	10.13 ± 0.01	10.11 ± 0.03
PDW (fL)	11.65 ± 0.02	11.35 ± 0.02	11.36 ± 0.06
PCT (%)	0.34 ± 0.01	0.31 ± 0.00	0.34 ± 0.00
RDW-CV (%)	14.13 ± 0.01	14.33 ± 0.02	14.62 ± 0.05
TP (g/L)	69.53 ± 0.05	71.35 ± 0.08	70.50 ± 0.26
ALB (g/L)	45.07 ± 0.03	44.88 ± 0.05	43.73 ± 0.16
GLB (g/L)	24.45 ± 0.04	26.47 ± 0.07	26.77 ± 0.22
ALB/GLB	1.92 ± 0.00	1.78 ± 0.01	1.73 ± 0.01
PA (mg/L)	154.07 ± 0.32	158.10 ± 0.43	154.12 ± 1.16
TBIL (*μ*mol/L)	7.17 ± 0.04	7.41 ± 0.04	6.69 ± 0.10
DBIL (*μ*mol/L)	2.48 ± 0.01	2.63 ± 0.02	2.43 ± 0.05
IDBL (*μ*mol/L)	4.70 ± 0.04	4.79 ± 0.03	4.26 ± 0.07
ALT (U/L)	24.10 ± 0.29	22.93 ± 0.36	24.49 ± 1.14
AST (U/L)	47.20 ± 0.24	45.40 ± 0.28	49.48 ± 1.53
AST/ALT	2.38 ± 0.01	2.42 ± 0.01	2.50 ± 0.06
ALP (U/L)	217.48 ± 1.20	226.55 ± 1.96	214.66 ± 4.18
GGT (U/L)	12.50 ± 0.10	13.98 ± 0.14	15.33 ± 0.43
5-NT (U/L)	5.31 ± 0.03	5.23 ± 0.04	5.04 ± 0.08
LDH (U/L)	426.74 ± 1.18	447.45 ± 1.69	463.15 ± 6.15
CK (U/L)	159.37 ± 3.22	154.94 ± 2.24	201.86 ± 11.10
CK-MB (U/L)	20.34 ± 0.13	17.02 ± 0.15	17.86 ± 0.39
CK/CK-MB	8.78 ± 0.08	10.80 ± 0.13	12.12 ± 0.43
CnTI (ng/mL)	0.49 ± 0.01	0.48 ± 0.01	0.49 ± 0.01
Mb (*μ*g/L)	26.49 ± 0.28	22.04 ± 0.30	53.02 ± 3.22
*β*2MG (mg/L)	2.51 ± 0.01	2.31 ± 0.01	2.15 ± 0.02
CRP (mg/L)	19.50 ± 0.20	12.99 ± 0.21	10.82 ± 0.47
SAA (mg/L)	22.30 ± 0.08	23.48 ± 0.11	23.31 ± 0.29
Glu (mmol/L)	4.44 ± 0.01	5.08 ± 0.02	5.74 ± 0.07
BUN (mmol/L)	3.80 ± 0.01	3.58 ± 0.01	3.69 ± 0.05
CR (*μ*mol/L)	27.57 ± 0.07	28.72 ± 0.15	29.40 ± 0.37
BUN/CR	0.15 ± 0.00	0.13 ± 0.00	0.13 ± 0.00
UA (*μ*mol/L)	264.84 ± 0.78	263.40 ± 1.10	275.28 ± 4.01
K (mmol/L)	4.62 ± 0.01	4.57 ± 0.01	4.46 ± 0.02
Ca (mmol/L)	2.45 ± 0.00	2.45 ± 0.00	2.42 ± 0.00
Na (mmol/L)	139.23 ± 0.03	138.40 ± 0.04	137.93 ± 0.11
Mg (mmol/L)	0.97 ± 0.00	0.97 ± 0.00	0.97 ± 0.00
Cl (mmol/L)	104.79 ± 0.03	103.22 ± 0.04	102.51 ± 0.11
P (mmol/L)	1.64 ± 0.00	1.62 ± 0.00	1.62 ± 0.01

Note: values were presented with mean ± SEM. SP: systolic pressure; DP: diastolic pressure; NEUT#: neutrophil count; NEUT%: neutrophil ratio; LYMPH#: lymphocyte count; LYMPH%: lymphocyte ratio; MONO#: mononuclear cell; MONO%: mononuclear cell ratio; EO#: eosinophil; EO%: eosinophil ratio; BASO#: basophils; BASO%: basophil ratio; WBC: white blood cell; RBC: red blood cell; HGB: hemoglobin; MCH: mean corpuscular hemoglobin; MCHC: mean corpuscular hemoglobin concentration; RDW-SD: red blood cell distribution width; HCT: hematocrit; MCV: mean corpuscular volume; PLT: platelet; P-LCR: platelet-large cell ratio; MPV: mean platelet volume; PDW: platelet distribution width; PCT: thrombocytocrit; TP: total protein; ALB: albumin; GLB: globulin; PA: prealbumin; TBIL: total bilirubin; DBIL: direct bilirubin; IDBL: indirect bilirubin; ALT: glutamic-pyruvic transaminase; AST: glutamic oxalacetic transaminase; ALP: alkaline phosphatase; GGT: gamma-glutamyl transferase; 5-NT: 5′-nucleotidase; LDH: lactate dehydrogenase; CK: creatine kinase; CK-MB: creatine kinase-myocardial band isoenzyme; CnTI: cardiac troponin; Mb: myohemoglobin; CRP: c-reaction protein; SAA: serum amyloid A; Glu: glucose; BUN: urea; CR: creatinine; UA: uric acid; K: potassium; Ca: calcium; Na: sodium; Mg: magnesium; Cl: chlorine; P: phosphorus.

The article "Development and Validation of Diagnostic Models for Hand-Foot-and-Mouth Disease in Children" was retracted in 2023. Reasons: unreliable results or conclusions; concerns about the data; concerns about the peer review; concerns about the citations.

**Table 2:** Difference indexes and fold change (FC) value.

Characteristics	Mild vs. severe		Mild vs. severe-RF		Severe vs. severe-RF	
	*P*	FC	*P*	FC	*P*	FC
SP	∗∗∗	1.04	∗∗∗	1.10	∗∗∗	1.07
DP	∗∗∗	1.06	∗∗∗	1.12	∗∗∗	1.06
NEUT#	∗∗∗	1.07	∗∗∗	1.35	∗∗∗	1.27
NEUT%	∗∗∗	1.11	∗∗∗	1.24	∗∗∗	1.11
RDW-SD	∗∗∗	1.02	∗∗∗	1.04	∗∗∗	1.02
RDW-CV	∗∗∗	1.01	∗∗∗	1.03	∗∗∗	1.02
GGT	∗∗∗	1.12	∗∗∗	1.23	∗∗	1.10
LDH	∗∗∗	1.05	∗∗∗	1.09	∗	1.04
CK/CK-MB	∗∗∗	1.23	∗∗∗	1.38	∗∗	1.12
Glu	∗∗∗	1.14	∗∗∗	1.29	∗∗∗	1.13
LYMPH%	∗∗∗	0.90	∗∗∗	0.77	∗∗∗	0.86
MONO%	∗∗∗	0.84	∗∗∗	0.72	∗∗∗	0.86
EO#	∗∗∗	0.50	∗∗∗	0.33	∗∗∗	0.67
EO%	∗∗∗	0.44	∗∗∗	0.26	∗∗∗	0.59
BASO%	∗∗∗	0.87	∗∗∗	0.60	∗∗∗	0.69
MCHC	∗∗∗	0.99	∗∗∗	0.99	∗∗∗	0.99
ALB/GLB	∗∗∗	0.93	∗∗∗	0.90	∗∗	0.97
*β*2MG	∗∗∗	0.92	∗∗∗	0.86	∗∗∗	0.93
CRP	∗∗∗	0.67	∗∗∗	0.55	∗∗∗	0.83
K	∗∗∗	0.99	∗∗∗	0.97	∗∗∗	0.98
Cl	∗∗∗	0.99	∗∗∗	0.98	∗∗∗	0.99
Na	∗∗∗	0.99	∗∗∗	0.99	∗∗∗	0.99
ALB	∗∗	0.98	∗∗∗	0.97	∗∗∗	0.97
BASO#	∗∗∗	1.00	∗∗∗	0.50	∗∗	0.50
WBC	∗∗∗	0.97	∗∗∗	1.12	∗∗∗	1.15
TP	∗∗∗	1.03	∗∗∗	1.01	∗∗	0.99
TBIL	∗∗	1.03	∗∗	0.93	∗∗∗	0.90
CK-MB	∗∗∗	0.84	∗∗∗	0.88	∗	1.05
Mb	∗∗∗	0.83	∗∗∗	2.00	∗∗∗	2.41
BUN	∗∗∗	0.94	∗	0.97	∗	1.03
Age	-	-	-	-	∗	-
Gender	-	-	∗	-	-	-
Temperature	∗∗∗	1.02	∗∗∗	1.02	-	-
LYMPH#	∗∗∗	0.90	∗∗∗	0.88	-	-
MONO#	∗∗∗	0.81	∗∗∗	0.78	-	-
RBC	∗∗∗	1.01	∗	1.01	-	-
HGB	-	-	∗∗∗	0.98	∗∗∗	0.98
MCH	-	-	∗∗	0.99	∗∗	0.99
HCT	∗∗∗	1.01	-	-	∗	0.99
MCV	∗∗∗	1.01	-	-	-	-
PLT	-	-	∗∗∗	1.10	∗∗∗	1.10
P-LCR	∗∗∗	0.95	∗∗∗	0.95	-	-
MPV	∗∗∗	0.98	∗∗∗	0.98	-	-
PDW	∗∗∗	0.97	∗∗∗	0.98	-	-
PCT	∗∗∗	0.91	-	-	∗∗∗	1.10
GLB	∗∗∗	1.08	∗∗∗	1.09	-	-
PA	∗∗∗	1.03	-	-	∗∗	0.97
DBIL	∗∗∗	1.06	-	-	∗∗∗	0.92
IDBL	-	-	∗∗	0.91	∗∗∗	0.89
ALT	∗	0.95	-	-	-	-
AST	∗∗∗	0.96	-	-	∗∗	1.09
AST/ALT	∗	1.02	-	-	-	-
ALP	∗∗∗	1.04	-	-	∗	0.95
5-NT	-	-	∗∗	0.95	-	-
CK	-	-	∗∗∗	1.27	∗∗	1.30
SAA	∗∗∗	1.05	∗∗	1.05	-	-
CR	∗∗∗	1.04	∗∗∗	1.07	-	-
BUN/CR	∗∗∗	0.87	∗∗∗	0.87	-	-
UA	-	-	∗	1.04	∗∗	1.05
Ca	-	-	∗∗∗	0.99	∗∗∗	0.99
P	∗∗∗	0.99	∗	0.99	-	-

∗∗∗, ∗∗, and ∗: *P* < 0.001, 0.01, and 0.05, respectively; “-” represents the statistical significance of *P* values more than 0.05.

**Table 3:** Top 10 indicators of AUROC value in each group.

Mild vs. severe			Mild vs. severe-RF			Severe vs. severe-RF		
	AUROC	95% CI		AUROC	95% CI		AUROC	95% CI
Temperature	0.74	0.74-0.75	Glu	0.80	0.78-0.82	Glu	0.68	0.66-0.70
EO#	0.69	0.68-0.70	EO%	0.75	0.74-0.77	Ca	0.66	0.64-0.68
Glu	0.69	0.68-0.70	EO#	0.75	0.73-0.77	SP	0.65	0.63-0.67
EO%	0.68	0.68-0.69	SP	0.74	0.72-0.76	*β*2MG	0.65	0.63-0.66
Cl	0.65	0.65-0.66	Temperature	0.73	0.71-0.75	Mb	0.63	0.61-0.65
*β*2MG	0.64	0.63-0.65	Cl	0.71	0.69-0.73	NEUT#	0.62	0.60-0.64
MONO%	0.63	0.62-0.64	*β*2MG	0.71	0.69-0.72	NEUT%	0.61	0.59-0.63
SP	0.62	0.62-0.63	MONO%	0.70	0.69-0.72	LYMPH%	0.61	0.59-0.63
CK-MB	0.61	0.60-0.62	NEUT%	0.70	0.69-0.72	PCT	0.59	0.57-0.61
NEUT%	0.61	0.60-0.62	DP	0.68	0.66-0.70	DP	0.59	0.57-0.61

## Data Availability

The data used to support the findings of this study are included within the article.

## References

[1] Qin L., Dang D., Wang X. (2019). Identification of immune and metabolic predictors of severe hand-foot-mouth disease. *PLoS One*.

[2] Dolin R. (1999). Enterovirus 71 — Emerging infections and emerging questions. *The New England Journal of Medicine*.

[3] Zhang S. Y., Xu M. Y., Xu H. M. (2015). Immunologic characterization of cytokine responses to enterovirus 71 and coxsackievirus A16 infection in children. *Medicine (Baltimore)*.

The article "Development and Validation of Diagnostic Models for Hand-Foot-and-Mouth Disease in Children" was retracted in 2023. Reasons: unreliable results or conclusions; concerns about the data; concerns about the peer review; concerns about the citations.

[4] Leung G. M., Xing W. J., Wu J. T., Yu H. (2014). Hand, foot, and mouth disease in mainland China-Authors' reply. *Lancet Infectious Diseases*.

[5] Van Voorhis K. T., Willis T. S. (2009). Implementing a pediatric rapid response system to improve quality and patient safety. *Pediatric Clinics of North America*.

[6] Monaghan A. (2005). Detecting and managing deterioration in children. *Paediatric Nursing*.

[7] Wang B., Feng H., Huang P. (2019). Developing a nomogram for risk prediction of severe hand-foot-and-mouth disease in children. *Indian Journal of Pediatrics*.

[8] Liu C., Wang K., Lin N., Cai J., Cui B., Wu B. (2018). Risk factors of severe hand, foot and mouth disease in Shantou, China: a case-control study. *Journal of Infection in Developing Countries*.

[9] Ni X. F., Li X., Xu C. (2020). Risk factors for death from hand-foot-mouth disease: a meta-analysis. *Epidemiology and Infection*.

[10] Mei L., Song X., Kong Y., Yu G. (2018). An assessment of a pediatric early warning system score in severe hand-foot-and-mouth disease children: to detect clinical deterioration in hospitalized children. *Medicine (Baltimore)*.

[11] Schisterman E. F., Faraggi D., Reiser B., Trevisan M. (2001). Statistical inference for the area under the receiver operating characteristic curve in the presence of random measurement error. *American Journal of Epidemiology*.

[12] Bozdogan H. (2000). Akaike's Information Criterion and Recent Developments in Information Complexity. *Journal of Mathematical Psychology*.

[13] Sun B. J., Chen H. J., Chen Y., An X. D., Zhou B. S. (2018). The Risk Factors of Acquiring Severe Hand, Foot, and Mouth Disease: A Meta- Analysis. *Canadian Journal of Infectious Diseases and Medical Microbiology,*.

[14] Peng L., Luo R., Jiang Z. (2017). Risk factors for neurogenic pulmonary edema in patients with severe hand, foot, and mouth disease: a meta-analysis. *International Journal of Infectious Diseases*.

[15] Fang Y., Wang S., Zhang L. (2014). Risk factors of severe hand, foot and mouth disease: a meta-analysis. *Scandinavian Journal of Infectious Diseases*.

[16] Lin H., Zou H., Wang Q. (2013). Short-term effect of El Niño-Southern Oscillation on pediatric hand, foot and mouth disease in Shenzhen, China. *PLoS One*.

[17] Feng H., Duan G., Zhang R., Zhang W. (2014). Time series analysis of hand-foot-mouth disease hospitalization in Zhengzhou: establishment of forecasting models using climate variables as predictors. *PLoS One*.

[18] Li L., Qiu W., Xu C., Wang J. (2018). A spatiotemporal mixed model to assess the influence of environmental and socioeconomic factors on the incidence of hand, foot and mouth disease. *BMC Public Health*.

The article "Development and Validation of Diagnostic Models for Hand-Foot-and-Mouth Disease in Children" was retracted in 2023. Reasons: unreliable results or conclusions; concerns about the data; concerns about the peer review; concerns about the citations.

[19] Grady D., Berkowitz S. A. (2011). Why is a good clinical prediction rule so hard to find?. *Archives of Internal Medicine*.

[20] Liu G., Xu Y., Wang X. (2017). Developing a machine learning system for identification of severe hand, foot, and mouth disease from electronic medical record data. *Scientific Reports*.

